# Application Value of the Workshop Practice Teaching Method Based on Target-Oriented Study Modules on the Internet in Orthopedic Rehabilitation

**DOI:** 10.1155/2022/5166219

**Published:** 2022-01-27

**Authors:** Qian He, Guanqun Ge, Qiong Wu, Yanchao Cui

**Affiliations:** ^1^Student Work Office of the First Affiliated Hospital of Xi'an Jiaotong University, Xi'an City 710061, Shaanxi Province, China; ^2^Department of Breast Surgery of the First Affiliated Hospital of Xi'an Jiaotong University, Xi'an City 710061, Shaanxi Province, China; ^3^Department of Rehabilitation Medicine of the First Affiliated Hospital of Xi'an Jiaotong University, Xi'an City 710061, Shaanxi Province, China

## Abstract

**Objective:**

To explore the application value of the workshop practice teaching method based on target-oriented study modules on the internet in orthopedic rehabilitation.

**Methods:**

Thirty interns (2019-2020) in the rehabilitation department of our hospital were selected as the control group, another thirty interns (2021) in the rehabilitation department of our hospital were selected as the experimental group, and their materials were retrospectively reviewed. Both groups were given the three-month practice teaching. Besides, the conventional practice teaching method was applied to the control group, and the workshop practice teaching method based on target-oriented study modules on the internet was applied to the experimental group. After the practice teaching, the united examination paper and assessment table of the rehabilitation operation process were used to evaluate the interns' scores of theoretical knowledge about orthopedic rehabilitation, scores of practical skills, and comprehensive scores of clinical practice in the two groups. The evaluation team consisting of 5 guiding experts in the scientific research office assessed the teaching quality of the two methods.

**Results:**

Compared with the control group, the experimental group had a notably higher score of theoretical knowledge about orthopedic rehabilitation, higher score of practical skills, and higher comprehensive score of clinical practice (92.47 ± 4.81 vs. 86.43 ± 5.12, 91.30 ± 5.68 vs. 81.53 ± 7.21, and 91.88 ± 2.45 vs. 83.98 ± 4.42, *P* < 0.001). According to the evaluation team, the teaching quality of the experimental group was observably higher than that in the control group (*P* < 0.05), and there was no remarkable difference in the scores of teachers' performance between the two groups (*P* > 0.05).

**Conclusion:**

The workshop practice teaching method based on target-oriented study modules on the internet, as a high-quality “Internet+” practice teaching mode, can improve the orthopedic interns' scores of theoretical knowledge and practical operation ability and enhance their comprehensive qualities of orthopedic rehabilitation in all respects.

## 1. Introduction

Orthopedic rehabilitation refers to adopting the measures such as physiotherapy and exercise therapy to speed up the recovery of somatic motor functions and reduce the degree of limb function damage, thus enabling the patients to successfully return to the normal life. At present, with the changes of Chinese people's lifestyle, the incidence of orthopedic diseases has shown an increasing trend [1], and the clinical requirements for orthopedists are even higher than before. As the orthopedics is a highly specialized clinical discipline, orthopedists should possess both theoretical knowledge and practical skills. Especially under the background where the medical field develops rapidly, the orthopedists must constantly improve their skills and master theoretical knowledge in depth to meet the needs of practice. The scientific practice teaching measures are important for the orthopedic interns to successfully become the qualified orthopedists. During their internship, the interns can fully apply their knowledge and theories in practice, accumulate clinical experience, and improve their comprehensive qualities [2, 3]. In order to achieve the goal of cultivating orthopedic talents in all aspects, it is necessary to continuously optimize the practice teaching measures in clinics, fully absorb the advanced practice teaching experience at home and abroad, and apply the excellent educational concepts in orthopedic practice teaching. With the further development of orthopedic rehabilitation treatment in recent years, the guided and heuristic practice teaching methods have been introduced into China [4, 5], and its representative is the workshop practice teaching method, which takes the students as the core of education, aims at developing the students' professional and practical skills, and improves their qualities in practice to avoid the empty teaching. The modules of employable skills (MES) offer a sound basis to the modular teaching of the workshop because the workshop aims at skill training. The MES prioritize on-the-spot teaching, take skill training as the core of education, and focus on postcompetency [6]. With the rise of internet medicine, there is more extensive development space for the MES teaching mode. A large number of studies have shown that the “Internet+” platform can improve the effectiveness of clinicians and nursing staff [7, 8], so the “Internet+” target-oriented study module may further enhance the teaching quality of the workshop and make the training of orthopedic interns meet the developing requirements of orthopedic rehabilitation in practice.

Therefore, 30 orthopedic interns were given the workshop practice teaching method based on target-oriented study modules on the internet in this study, with the results summarized as follows.

## 2. Materials and Methods

### 2.1. Study Design

This was a retrospective study and conducted in our hospital from 2019 to 2021 to explore the application value of the workshop practice teaching method based on target-oriented study modules on the internet in orthopedic rehabilitation.

### 2.2. General Data

Thirty interns (2019-2020) in the rehabilitation department of our hospital were selected as the control group, and another thirty interns (2021) in the rehabilitation department of our hospital were selected as the experimental group. All the interns were undergraduates and were taught by 6 tutors, who were the senior doctors and therapists specializing in orthopedic rehabilitation with bachelor degree or above and with more than 3 years of practice teaching experience. In the experimental group, there were 18 males and 12 females with a mean age of 24.40 ± 1.56 years. In the control group, there were 19 males and 11 females with a mean age of 24.37 ± 1.38 years. No statistical difference in the interns' general data (such as age and sex ratio) between the two groups was observed (*P* > 0.05), and the interns in the two groups could be taken as the study subjects.

### 2.3. Steps

The total 60 interns in the rehabilitation department in this study were divided into the experimental group and control group according to their internship time. The conventional practice teaching method was applied to the control group. The workshop practice teaching method based on target-oriented study module on the internet was applied to the experimental group. The united examination paper and assessment table of the rehabilitation operation process were used to evaluate the interns' scores of theoretical knowledge about orthopedic rehabilitation, scores of practical skills, and comprehensive scores of clinical practice of the two groups after the internship. The evaluation team consisting of 10 guiding experts in the scientific research office evaluated the teaching quality of the two methods.

### 2.4. Moral Consideration

The study was performed in accordance with the principles of Declaration of Helsinki (2013) [9], and all the interns agreed to participate in the study.

### 2.5. Methods

The conventional practice teaching method was applied to the control group. One tutor was in charge of six interns. The tutors took the interns to conduct teaching ward rounds and organize discussions on typical cases, which could inspire the interns' clinical thought, cultivate their ability to recognize, analyze, and solve problems, and enable them to gradually acquire the important knowledge of orthopedic rehabilitation and meet the task requirements of the syllabus set by the scientific research office. The tutors should also conduct small clinical lectures to gradually cultivate the interns' writing ability and thinking of medical documents, instruct them to conduct inquisitions and physical examinations, and write medical records.

The experimental group received the workshop practice teaching method based on target-oriented study modules on the internet. (1) The platform of “Internet+” practice teaching was established, and different functional parts were designed in the platform according to the practice requirements of orthopedic rehabilitation. The comprehensive, independent, open, and flexible study modules were formed, and each module corresponded to one learning target. (2) As soon as the interns entered the group, they established archives of themselves and brought the group members into the established practice teaching group of orthopedic rehabilitation. The online study group was formed, and the interns collectively learned how to use the practice teaching platform of orthopedic rehabilitation and got familiar with the learning targets of each module. Six tutors were jointly in charge of 30 interns, and they had clear division of work according to the teaching targets. They carried out teaching tasks based on the “Internet+” teaching modules. (3) The workshop practice teaching was carried out in the platform of “Internet+” practice teaching, which meant that the workshop teaching was conducted based on the functional modules, and every special lecture, clinic instruction, and practical operation corresponded to the functional modules. (4) The preview module was mainly used for preclass learning. The tutors prepared 5 or 6 knowledge points related to the orthopedic rehabilitation and provided corresponding learning links for the interns to learn in advance by reviewing the literature. The module of special lectures contained new technologies and knowledge of orthopedics so that the interns could keep abreast of the new developments of medicine at home and abroad and increase their scientific research awareness during the learning. During the offline teaching, the interns could talk about the contents of the special lectures and think about the combination of the contents and existing technologies. The tutors summarized and commented on the interns' opinions. The module of theoretical study focused on the theoretical knowledge, including the secondary modules of muscle strength training, joint proprioception, gait training, joint function training, rehabilitation treatment of neurological function, and balance function training. After the teaching, the tutors made class summaries and entered the plain text version of the knowledge into the platform, facilitating interns' review after class. The module of classroom test was formulated by the tutors according to the task requirements in the syllabus and included the theoretical knowledge module and practice module. Both modules were subdivided into the secondary modules of muscle strength training, joint proprioception, gait training, joint function training, rehabilitation treatment of neurological function, balance function training, and so on. The in-class assessment of theoretical knowledge was conducted in each secondary module in the manner of online questionnaires. The in-class assessment of practical skills was conducted in offline teams. The interns should well digest and completely understand the theoretical knowledge, apply it into practice flexibly, and avoid the rote learning. This module sufficiently investigated the interns' mastery of the orthopedic rehabilitation measures and their application ability of these measures.

### 2.6. Evaluation Criteria

1. Assessment scores: ① assessment of theoretical knowledge: the teaching and research office drew up an examination paper according to the syllabus and the actual teaching situation, and the interns took the closed-book exam at the end of the internship. The exam time was 120 minutes, and the scores were 0–100 points. ② Assessment of practical skills: the assessment of practical skills was conducted in the orthopedic rehabilitation training room, with one tutor playing the patient and one tutor monitoring the exam. The evaluation team consisting of 5 guiding experts in the scientific research office adopted the united assessment table of the rehabilitation operation process to give scores (0–100 points) to the interns according to the standardization, accuracy, and completion of their operation. ③ The comprehensive score of clinical practice: the comprehensive score = (the score of theoretical knowledge + the score of practical skills)/2.
2. Teaching quality: during the study of the interns in the two groups, the evaluation team randomly selected 5 lessons for scoring the teaching quality. The scoring items included teaching facility (the teaching facility in the experimental group included the platform of “Internet+” practice teaching), case study, group cooperation, teachers' performance, teacher-student interaction, class design, teaching effect, and cultivation of critical thinking, with 0–10 points for each item. Higher scores represented higher teaching quality.

### 2.7. Statistical Treatment

This study adopted SPSS 20.0 as data processing software and GraphPad Prism 7 (GraphPad Software, San Diego, USA) as graph drawing software. The study included count data and measurement data and used *X*^2^ test and *t*-test. When *P* < 0.05, the differences were considered statistically significant.

## 3. Results

### 3.1. Comparison of the Interns' Scores

Compared with the control group, the assessment scores of the experimental group were notably higher (*P* < 0.001; Figure 1).

Compared with the control group, the experimental group had a notably higher score of theoretical knowledge about orthopedic rehabilitation, higher score of practical skills, and higher comprehensive score of clinical practice (92.47 ± 4.81 vs. 86.43 ± 5.12, 91.30 ± 5.68 vs. 81.53 ± 7.21, and 91.88 ± 2.45 vs. 83.98 ± 4.42, *P* < 0.001).

### 3.2. Comparison of the Teaching Quality of the Two Practice Teaching Methods

According to the evaluation team, the teaching quality in the experimental group was observably higher than that in the control group (*P* < 0.05), and there was no remarkable difference in the scores of teachers' performance between the two groups (*P* > 0.05; Table 1).

## 4. Discussion

The orthopedic rehabilitation, as an important aspect of orthopedic treatment, has strong practicality and theoretical characteristic. Therefore, the clinical teaching of orthopedic rehabilitation should place emphasis on the interns' thorough digestion and complete understanding of the theoretical knowledge, so as to improve their clinical application ability in all respects [10–12]. At present, most practice teaching of orthopedic rehabilitation in China still adopts the traditional mode, which is tutor-centred. Under this mode, the students learn knowledge and solidify their memories for theories mainly through the tutors' classroom lectures. Although this practice teaching method can increase the interns' knowledge, it cannot arouse their learning enthusiasm, and interns cannot fully apply the theoretical knowledge in practice and enhance their practical operation ability. In recent years, with the continuous development of medical technology and increased demands for refined rehabilitation in clinics, the excellent practice teaching modes related to rehabilitation treatment have been gradually introduced into China [13–16]. Among these teaching modes, the workshop teaching method is one of the typical heuristic and interactive teaching modes and has been preliminarily applied in the teaching of some disciplines. The workshop teaching method is different from the traditional practice teaching method which takes the tutor's lecture as the core and divides the teaching contents into different modules. This teaching method aims at developing the professional and practical skills of the students, guides them to learn in practice, and avoids the overtheoretical teaching contents [17–19], so as to accelerate the development of their personal ability. According to the study of scholars Sitobata and Mohammadnezhad, the workshop teaching method is conducive to enhancing team cohesion and collaboration, improving the efficiency of teacher-student communication, and breaking communication barriers [20]. As the country vigorously advocates “Internet+” intelligent medical treatment, the workshop teaching method is facing the opportunity for innovation. If the project-based workshop teaching method can be perfectly combined with the “Internet+” modular teaching mode, it will become an advanced teaching mode with contemporary characteristics.

The “Internet+” modular teaching refers to the modular teaching based on the internet [7]. The modular teaching originates from the vocational education in European and American countries, and the competency-based education (CBE) mode and MES mode have become popular in China at present. The former focuses on the vocational ability training and the latter on the professional skill training [21]. Compared with the CBE mode, the MES mode adopted in this study more complies with the requirements of orthopedic rehabilitation in practice [22–24]. Besides, there is good synergy between the MES mode and the workshop teaching method, both of which aim to enhance the interns' professional skills through the modular (project-based) teaching. Through different modules on the platform of “Internet+” practice teaching, the interns could better practice the independent learning concept (advocating active exploration and automatic learning) of the workshop and take the initiative to expand learning contents around the teaching targets. This teaching method helps the interns to clearly understand the learning task in each lesson, and they could preview and review the lessons and take quizzes according to the tasks in the module. By combining the knowledge learned online with the offline group discussion, group cooperation, and teacher lectures, this teaching method takes the dual advantages of the online + offline teaching. According to the evaluation team, the teaching quality in the experimental group was observably higher than that in the control group after the systematic practice teaching (*P* < 0.05), which indicated that the workshop practice teaching method based on target-oriented study modules on the internet could improve the practice teaching quality with diversified teaching forms and systematized teaching results, so the interns in the experimental group had better participatory experience and deeper understanding of the knowledge they had learned. Therefore, the examination scores of the experimental group were markedly higher compared with the control group (*P* < 0.001), indicating that this teaching method could effectively link the theory with practice.

In conclusion, there are still many problems in the practice teaching of orthopedic rehabilitation at present, and it is necessary to explore more advanced practice teaching methods. According to this study, the workshop practice teaching method based on target-oriented study modules on the internet, as a high-quality “Internet+” practice teaching mode, can improve the orthopedic interns' scores of theoretical knowledge and practical operation ability and enhance their comprehensive abilities in the orthopedic rehabilitation to meet the requirements of clinical rehabilitation.

## Figures and Tables

**Figure 1:** Comparison of the interns' scores ($\bar{x}\pm s$, points). (a) Scores of theoretical knowledge. (b) Scores of practical skills. (c) Comprehensive scores of clinical practice.

**Table 1:** Comparison of the teaching quality of the two practice teaching methods ($\bar{x}\pm s$, points).

Group	Teaching facility	Case study	Group cooperation	Teachers' performance	Teacher-student interaction	Class design	Teaching effect	Cultivation of critical thinking
Experimental group	8.80 ± 0.75	9.00 ± 1.10	9.80 ± 0.40	9.20 ± 0.75	9.40 ± 0.49	9.20 ± 0.75	9.40 ± 0.80	9.00 ± 0.63
Control group	6.80 ± 1.72	7.40 ± 1.02	7.40 ± 1.02	9.00 ± 1.10	7.80 ± 1.17	7.60 ± 1.02	7.80 ± 0.75	7.60 ± 1.02
*t*	2.383	2.384	4.898	0.336	2.821	2.826	3.263	2.611
*P*	0.044	0.044	0.001	0.746	0.022	0.022	0.012	0.031

## Data Availability

The data used to support the findings of this study are available from the corresponding author upon reasonable request.
